# Predictors of Physical Activity Behavior Transitions in Children and Adolescents: A Systematic Review Based on a Transtheoretical Model

**DOI:** 10.1155/2023/5786841

**Published:** 2023-02-14

**Authors:** Jie Sheng, Peng Shi, Jinyue Sun, Xiaosu Feng

**Affiliations:** ^1^School of Art, Qingdao University of Science and Teachnology, Qingdao, China; ^2^School of Physical Education, Shanghai University of Sport, Shanghai, China; ^3^School of Physical Education, Liaoning Normal University, Dalian, China

## Abstract

**Background:**

The transtheoretical model (TTM) views individual behavioral change as a nonlinear, dynamic process, which is consistent with the complex nature of physical activity (PA) in children and adolescents. However, within this theoretical framework, the elements that facilitate the behavioral change in PA in children and adolescents need to be further explored.

**Objective:**

A systematic review of research related to TTM-based exploration of the elements of behavioral change in PA in children and adolescents, an analysis of the strengths and weaknesses in practice, and an outlook for future research.

**Materials and Methods:**

After computer searches of the CNKI, Wan-Fang, VIP, WOS, PubMed, and EBSCO databases, two researchers independently screened articles, extracted information, and evaluated the quality of the articles.

**Results:**

A total of 25 articles (26 studies) of medium- to high-quality were included in the systematic review. The meta-analysis included 30,106 children and adolescents aged 11.24 to 17.7 years. The counter-conditioning and self-liberation of the process of change, self-efficacy and decisional balance are key elements that facilitate the transition of the PA stage in children and adolescents. Extramodel psychological variables such as exercise motivation play a moderate to large role in the PA stage transition. In addition, VPA is an important discriminator of PA stage transition in children and adolescents.

**Conclusion:**

It is recommended that interventions be designed according to the key elements of behavioral change in order to better facilitate the PA stage transition of children and adolescents.

## 1. Introduction

Physical activity (PA) is any activity of the body that results from the contraction of skeletal muscles, leading to energy expenditure [1]. To date, numerous studies [2–5] have demonstrated that regular PA benefits children and adolescents in terms of cardiorespiratory endurance, mental health, cognitive function, and academic performance. Insufficient PA has become one of the four major risk factors for human death and is closely related to health problems such as obesity, hypertension, and diabetes in children and adolescents [6]. The World Health Organization (WHO) physical activity guidelines [7] recommend that school-age children and adolescents accumulate at least 60 min of moderate-to-vigorous physical activity (MVPA) per day. Despite the fact that the health benefits of PA have become common knowledge, the problem of inadequate PA in children and adolescents remains prominent and is gradually increasing with social changes [8, 9], making it imperative to develop effective PA promotion measures.

Exercise psychology provides many theoretical models for explaining, predicting, and intervening in PA behavior, among which the transtheoretical model (TTM) is considered to be a widely used stage model. Compared with other stage models such as the Health Action Process Approach (HAPA) and the Berlin Exercise Stage Model (BSM), TTM is more practical. TTM provides detailed change strategies to guide individuals at different stages of behavior change [10]. TTM has been widely used in health behavior research, such as on alcohol and drug abuse [11], eating disorders [12], physical exercise [13], and AIDS prevention [14]. TTM consists of four elements: the stage of change, the process of change, self-efficacy, and decisional balance (Figure 1; for a detailed description of TTM, see [10, 15, 16]).

TTM is well suited for exploring the PA behavior transition in children and adolescents. PA is behavior that includes participation in work, family, transportation, and recreational activities as a whole [17]. PA requires individuals to make balanced decisions based on the strengths and weaknesses of participating in PA and ultimately adapting to PA [18]. Because of the complexity of the PA transition, it requires a comprehensive theory to explain it. TTM, on the other hand, considers individual behavioral change as a nonlinear, dynamic process, which is linked to the complexity of PA. In addition, TTM has been shown to be effective in explaining and predicting PA behavioral changes in children and adolescents. Several studies [19, 20] have also shown that targeted intervention strategies based on TTM can help with individual stage promotion and PA improvement. Although TTM has accumulated a lot of research on the PA behavior transition of children and adolescents, its application is still questioned to varying degrees. The main reason for this is that there are so many components of the TTM [15]. The key predictors that influence the PA phase shift need to be further explored. So, what exactly are the factors that contribute to predicting the PA behavior transition in children and adolescents? How can the ability of TTM to explain PA changes in children and adolescents be further improved? No researcher has yet systematically analysed this. Based on this, the systematic reviews aim to identify the key predictors of PA behavior transition in children and adolescents, analyse the shortcomings, and make targeted recommendations. It is hoped that this will provide evidence to support the development of subsequent targeted intervention strategies.

## 2. Materials and Methods

### 2.1. Search Approach

In this study, Chinese and English search terms were used for literature searches. An electronic literature search was undertaken for articles published up to, and including, February 2022 on the online databases CNKI, Wan-Fang, VIP, Web of Science (WOS), PubMed, and EBSCO. Chinese search strategies: ((“跨理论模型 (TTM)” OR “变化阶段” OR “变化过程” OR “自我效能” OR “决策平衡”) AND (“身体活动” OR “体力活动” OR “锻炼” OR “久坐” OR “体质”)). English retrieval strategies: ((“transtheoretical model (TTM)” OR “stage of change” OR “process of change” OR “self-efficacy” OR “decisional balance”) AND (“physical activity” OR “exercise” OR “sedentary” OR “constitution” OR “physique”)).

### 2.2. Inclusion and Exclusion Criteria

Inclusion criteria for this study included (1) children and adolescents under 18 years of age; (2) TTM-based PA promotion; (3) crosssectional or longitudinal studies that examined the relationship between TTM components, other psychological variables, and PA; and (4) quantitative studies. Exclusion criteria for this study included (1) reviews, abstracts, comments, and letters; (2) literature not supported by accessible data; and (3) literature related to self-efficacy and decision-making balance not supported by TTM. In addition, for duplicate publications on the same study subject, only literature with complete studies was included. Two researchers independently screened the articles according to inclusion and exclusion criteria, in order of title, abstract, figure, and full text. The other two researchers conducted a secondary assessment, and, in case of dispute, a group discussion was held to decide jointly.

### 2.3. Quality Assessment

This study was assessed for quality using the STROBE statement [21], which consists of 22 items covering the title, abstract, introduction, methods, results, and discussion sections of the article. The STROBE statement provides guidance to researchers on how to improve the quality of observational studies and provides a methodological quality assessment tool for systematic reviews. Judgements based on the assessment tool are made independently by two researchers each, and where there are serious disagreements, entries are discussed with a third researcher.

## 3. Results

### 3.1. Results of the Search and Selection

A total of 10776 articles were retrieved, and another 6847 articles were obtained after being imported into the Endnote X9 software. Through literature selection, 25 articles were finally included. The literature selection process is shown in Figure 2.

### 3.2. Key Findings from a Study of Behavior Change in PA in Children and Adolescents

The year of publication for 25 papers was 1995 to 2021, with 1 of them [22] including 2 studies, resulting in a total of 26 studies being included (Table 1). A total of 30,106 children and adolescents from 14 countries were included. The sample size included in this study ranged from 244 to 5931, with a median of 819. The mean age of the subjects ranged from 11.24 to 17.7 years, and the percentage of females ranged from 35.8% to 100%. Twenty-three of the 26 studies were cross-sectional (88%), and three were longitudinal (12%). The quality of the included studies was rated as medium-high (15 to 21) with a median of 18. Stage algorithms for identifying PA change in children and adolescents included three types of forced-choice discrete measures (77%), progressive stage measures (19%), and scale continuous measures (4%). The main reasons for the lower quality rating were the failure to calculate the sample size, the failure to describe the subject recruitment method and sampling method, the failure to define criteria for regular PA at the stage of change, the failure to present statistics for judging predictive effects such as effect sizes and coefficients of determination, the failure to consider the effects of potential bias, and the failure to discuss the generalisability of the study results (external validity).

### 3.3. Predictors of PA Behavior Transition in Children and Adolescents

For cross-sectional studies exploring behavioral transitions in PA, *η*^2^ is commonly used to indicate the degree of contribution of factors. Therefore, this study judged the degree of effect of predictors based on Cohen's recommended effect sizes. If 0.01 ≤ *η*^2^ ≤ 0.06, it is a small effect size; if 0.07 ≤ *η*^2^ ≤ 0.14, it is a medium effect size; and if *η*^2^ > 0.14, it is a large effect size [47].

#### 3.3.1. The Process of Change

The process of change is the cognitive, emotional, and behavioral strategy that causes the transition in behavioral stages and is an important basis for developing intervention strategies. Burns et al. [41] found that, with increasing stage, Irish female adolescents showed a more positive process of change (*η*^2^ = 0.19). Which change strategies actually lead to behavioral transitions in children and adolescents with PA? The study sorted out the factors that achieved large effect sizes, including consciousness raising [24, 36], self-reevaluation [24], counter-conditioning [22, 24, 31, 36], helping relationships [24, 36], reinforcement management [24, 36], self-liberation [22, 24, 31, 36], and stimulus control [24, 36]. However, Bucksch et al. [37], Hwang, and Kim [39] showed that all change strategies had small effect sizes. The main reasons for this are the differences in the criteria for regular PA and the differences in the cross-cultural testing of the scales. What factors come into play during the adjacent stage transition? Wang et al. [27] found that cognitive processes play an important role in the process of behavioral intention enhancement and behavioral processes play an important role in the process of actual behavior facilitation. However, Fang [24] and Chen et al. [26] believed that the 10 dimensions of the process of change play different levels of importance in adjacent stages of transition and that there is not a strict correspondence between cognitive processes and behavioral intentions and behavioral processes and behavioral facilitation. It is important to note that dramatic relief and environmental reevaluation did not play any role in the adjacent stage of transition. Therefore, the relationship between the stage of change and the process of change needs to be further explored.

#### 3.3.2. Self-Efficacy and Decisional Balance

Diclemente et al. [48] introduced self-efficacy and decisional balance into the TTM to improve the model's predictive accuracy for phase transitions. Studies by De Bourdeaudhuij et al. [33] and Zamarripa et al. [43] have shown that decisional balance is a medium-to-large factor of effect for behavioral change in PA in children and adolescents. Several studies [23, 25, 32, 44, 45] have shown that there are stage differences in self-efficacy, positive benefits, and negative barriers, with self-efficacy and positive benefits increasing from the precontemplation to maintenance stages and negative obstacles decreasing. Numerous studies [22, 29, 34, 36, 41] have found that there are stage differences in both self-efficacy and decisional balance and that self-efficacy and positive benefits are medium to large effects and negative obstacles are medium-to-small effects. Reis and Petroski [35] and Abarca-Sos et al. [42] concluded that there are no gender differences in self-efficacy in PA behavioral change in Brazilian children and adolescents, whereas Abarca-Sos et al. [42] also found that internal obstacles acted to a greater extent for girls (*η*^2^ = 0.14) and external obstacles for boys (*η*^2^ = 0.04). All of the above studies showed that self-efficacy and decisional balance were predictors of behavioral change in children and adolescents with PA, but Bucksch et al. [37] showed no stage differences in negative barriers and small effect sizes for self-efficacy (*η*^2^ = 0.06) and positive benefits (*η*^2^ = 0.07).

#### 3.3.3. Other Psychological Variables

Some studies have explored the relationship of additional psychological variables to the PA stage transition in children and adolescents. This will help construct a factor set to better understand the pathways associated with the intervention and expand the theoretical framework of TTM. Related studies have demonstrated medium-to-large effects of exercise attitudes [33], exercise interests [41, 45], exercise motivation [25, 38, 44, 46], perceptual physical environment support [25, 41], perceptual social support [33, 41, 45], and physical self-concept [38, 41, 42] in the PA stage transition. Furthermore, Engels et al. [45] show that there are no stage differences in exercise knowledge, a view that appears to be contrary to common sense and needs to be further tested.

#### 3.3.4. PA Behavior Variables

The stage of change is a complex structure containing intentional, behavioral, and temporal components, and an increase in intention does not equal an increase in PA [40]. Behavioral factors are not only predictors of the stage of change in children and adolescents, but also discriminators of the effectiveness of testing stages [49]. Based on the concept of the stage of change, Hellsten et al. [50] suggested that there is a stage difference in PA with an increasing trend and proposed the hypothesis of “precontemplation/contemplation < preparation < action/maintenance” stages of PA. Abarca-Sos et al. [42] found that the physical activity index (PAI) was effective in distinguishing the stage of change and fully supported the hypothesis of the above study. However, some studies [33, 43] showed no significant difference in PA between the preparation and action stages; some studies [38, 45] also showed no significant difference in PA between the preparation and contemplation-forward (precontemplation and contemplation) stages. In addition, some studies [30, 33, 34] have shown that vigorous physical activity (VPA) has the highest differentiation, followed by moderate physical activity (MPA), with no stage differences in low-intensity physical activity (LPA).

### 3.4. Predictive Effects of PA Behavior Transition in Children and Adolescents

The focus of research in exercise psychology is to maximise the effectiveness of explanation and prediction of PA, to provide a theoretical framework for PA promotion, and thus to translate the available scientific evidence into practice. First, some studies have examined the predictive effect of psychological factors of TTM on behavioral transition in PA. Of these, the positive judgment rate for the PA stages of the process of change prediction was 47.4% [24]; self-efficacy and decision balance explain 40% of the variance in PA behavior change [23, 32]. Second, the predictive power of the model is enhanced by the addition of other factors to the original structure of the TTM. These factors mainly refer to PA behavior factors, and in particular, the VPA inclusion results in a positive judgement rate of over 60% [28, 34].

The chronological nature of the stages of change requires researchers to use more longitudinal studies to explore the antecedents of behavioral change over time, and unfortunately, there is a relative paucity of research in this area. Prapavessis et al. [22] explored the processes of change, self-efficacy, and decisional balance in predicting the PA stage transition of New Zealand adolescents at 6-month intervals. The results found the best predictions for counter-conditioning (*η*^2^ = 0.19), self-liberation (*η*^2^ = 0.15), and self-efficacy (*η*^2^ = 0.22), further supporting the cross-sectional study. The results of Nigg [31] showed that PA at baseline and self-efficacy were the most significant predictors of PA at follow-up for groups in the preparation, action, and maintenance phases (*R*^2^ = 0.31). Engels et al. [45] showed a low-to-moderate positive correlation between stage change and MVPA at 6-month intervals in Hawaiian children and adolescents. In addition, self-efficacy, exercise interest, family support, peer support, and exercise knowledge were less effective predictors of MVPA for boys (*R*^2^ = 0.139) and girls (*R*^2^ = 0.078).

In summary, the TTM and its extended model are effective in predicting the direction of PA behavior transition in children and adolescents. In addition, exploring the determinants and predictive effects of adjacent stage transitions is instructive for refining intervention strategies, but few studies have explored and tested this.

## 4. Discussion

This study is the first to explore the predictors of PA behavior change in children and adolescents based on TTM. It is the first to systematically examine the theoretical framework of TTM and helps provide a basis for the development of subsequent intervention strategies. As the stage of change rises, self-efficacy and positive benefits continue to increase and negative obstacles continue to decrease. The effect of self-efficacy and decisional balance on stage advancement is a medium-to-large effect, with a larger effect size for positive benefits and a smaller effect size for negative obstacles. However, differences in survey respondents, stage algorithms, and cultural differences led to large heterogeneity among similar studies, with only the large effects of counter-conditioning and self-liberation supported by the majority of the five studies that reported process-of-change effect sizes. In addition, extramodel psychological variables such as exercise motivation play a moderate-to-large role in the PA stage transition. For the behavioral factors, the association with the stages of change becomes stronger as the intensity of PA increases. The VPA can be effectively distinguished by the stage of change.

However, during the course of this review, this study found that there were still some shortcomings in TTM. First, the rationality of the division into stages of change has been questioned. There is a blurring of the concept of stages of change, particularly in the preparation phase. Some researchers [26, 28, and 31] have suggested that the preparation stage is one in which individuals have already attempted PA, just not on a regular basis. Some researchers [45, 51] also consider the preparation stage to be when the individual is not currently engaged in PA but is only making preparations to attend training, make plans, purchase equipment, etc., with the intention of making changes in the next 30 days. As a result, the PA is a poor predictor of the stage of change and does not fully support the “precontemplation/contemplation < preparation < action/maintenance” stage hypothesis. In addition, researchers often use PA to test the validity of the stage of change but are unable to distinguish between the precontemplation and contemplation stage and the action and maintenance stage. Second, the relationship between the structural elements within TTM is not yet clear. First, the relationship between the process of change and the stage of change has not yet led to a common conclusion. Repeated revisions of the process of change scale due to cultural differences are a major source of heterogeneity between studies. At the same time, environmental incentives are ignored as a component of self-efficacy. Although the field of health behavior has demonstrated an opposing relationship between environmental incentives and self-confidence [52], what environmental incentives are faced by children and adolescents with PA? How do environmental incentives predict changes in PA stages in children and adolescents? These questions have not yet been addressed. Finally, it has been pointed out that TTM is not applicable to PA, mainly because the real determinants of PA are not included in the model and it is difficult to predict the shift to specific stages of PA [53].

Based on these shortcomings, this study offers the following outlook for future studies: firstly, the concept of the stages of change still needs to be standardized and unified, and whether individuals in the preparation stage in particular engage in practical action requires further academic exploration. The stages of change can be compared across the different determination criteria by combining behavioral data, exercise intentions, and exercise habits. The concept and validity of the stages of change are tested on the basis of the hypothesis that behavioral data distinguish between physical activity and inactivity, exercise intentions between precontemplation and contemplation, and exercise habits between action and maintenance. Second, it is recommended that relevant researchers actively engage in academic exchanges, pool their ideas, unify their views, and compile appropriate measurement tools to better explore the relationship between the process of change and the stages of change. In addition, the construct of environmental incentives has not received much attention from researchers. It is recommended that follow-up studies explore the incentives of PA in children and adolescents through rooting theory, develop scales with high reliability and validity, and explore the role of environmental incentives in the stage transition to PA. Finally, the PA stage transition in children and adolescents is not fully explained; that is, TTM needs to be further developed and refined. The main approach to developing a theory is to integrate other variables. Behavior change theories have all received empirical support in practice, but each has also been challenged to varying degrees, so the integration of theoretical structures is seen as the way forward for behavior change theory [54].

## 5. Conclusion

This systematic review suggests that self-efficacy, decisional balance, and the counter-conditioning and self-liberation of the processes of change are key elements of behavioural change in PA in children and adolescents. In addition, VPA is an important discriminator of PA stage transition in children and adolescents. These findings provide psychological elements to support the development of subsequent PA promotion strategies for children and adolescents.

## Figures and Tables

**Figure 1:** Structure diagram of the transtheoretical model.

**Figure 2:** Literature selection flow chart.

**Table 1:** TTM-based studies on behavior change in PA in children and adolescents.

Included studies	Sample size	Nationality	Age	Woman (%)	Variables						Study design	Stage algorithm	Stage distribution (%)					Quality assessment
					SC	PC	SE	DB	PA	OV			PC	*C*	*P*	*A*	*M*	
Fang et al., [23]	1129	CHN	15.4	49.4	√		√	√			CSS	①	21.7	24.9	37.4	6.1	9.8	16
Fang, [24]	899	CHN	15.9 ± 1.3	56.0	√	√					CSS	①	3.0	20.8	51.1	14.0	11.1	19
Yi et al., [25]	1508	CHN	13.93 ± 1.00	50.5	√		√	√		√	CSS	①	8.1	9.7	47.7	16.3	18.1	16
Chen et al., [26]	430	CHN	11.24 ± 1.02	35.8	√	√	√	√			CSS	①	26.5	33.3	15.8	13.3	11.2	17
Wang et al., [27]	3000	CHN	11–17	48.4	√	√					CSS	③	14.8	22.4	32.2	17.6	13.0	17
Wyse et al., [28]	244	UK	17.7 ± 1.1	58.6	√		√		√	√	CSS	①	7.8	11.9	35.7	16.8	27.5	20
Nigg and Courneya [29]	819	CAN	15.0 ± 1.22	48.7	√	√	√	√			CSS	①	2.1	4.2	28.7	15.7	49.3	18
Lee et al., [30]	819	CAN	15.0 ± 1.2	49.0	√				√		CSS	①	2.1	4.2	28.7	15.7	49.3	17
Nigg, [31]	400	CAN	14.89 ± 1.15	54.8	√	√	√	√	√		LS	①	2.3	4.5	29.0	16.8	47.5	21
Prapavessis et al., [22]	3972	NZ	16.5 ± 0.76	53.4	√	√	√	√			CSS	①	6.2	8.7	40.8	19.2	25.0	20
Prapavessis et al., [22]	1434	NZ	16.41 ± 0.71	56.4	√	√	√	√			LS	①	N/A					19
Kim, [32]	671	KR	15.8	47.4	√		√	√			CSS	①	17.5	16.6	20.4	28.3	17.2	18
De Bourdeaudhuij et al., [33]	5931	BE	14.8 ± 1.9	61.0	√		√	√	√	√	CSS	②	11.5	16.0	13.8	8.3	50.4	20
Berry et al., [34]	311	CAN	15–17	43.4	√		√	√	√		CSS	①	1.9	6.1	23.8	16.4	51.8	19
Reis et al., [35]	488	BR	14–17	42.5	√		√		√	√	CSS	①	5.5	22.3	14.5	17.8	39.8	17
Sas-Nowosielski, [36]	1251	PL	17.33 ± 0.87	65.23	√	√	√	√			CSS	①	7.6	11.4	43.3	13.1	24.7	18
Bucksch et al., [37]	588	GER	15.0 ± 0.67	49.5	√	√	√	√			CSS	②	29.8	22.0	10.7	3.4	33.2	19
Parker et al., [38]	705	AUS	17.0 ± 0.96	52.0	√				√	√	CSS	②	4.0	7.0	13.0	6.0	70.0	16
Hwang and Kim, [39]	851	KR	16.0	43.7	√	√					CSS	①	25.2	27.3	13.7	15.8	18.0	16
Serra Puyal et al., [40]	831	ES	13.8 ± 1.4	54.3	√				√		CSS	①	2.3	6.9	34.0	12.2	44.6	16
Burns et al., [41]	871	IRL	15.28 ± 1.80	100	√	√	√	√		√	CSS	①	N/A					20
Abarca-Sos et al., [42]	1618	ES	14.46 ± 1.28	45.36	√		√	√	√	√	CSS	①	2.6	7.2	26.3	12.7	51.7	18
Zamarripa et al., [43]	285	MX	16.4 ± 1.3	57.5	√			√	√		CSS	②	7.7	37.2	13.7	10.9	30.5	15
Planas et al., [44]	372	ES	12–16	44.9	√			√		√	CSS	①	3.5	11.0	24.7	8.6	52.2	18
Engels et al., [45]	357	USA	14.24 ± 0.88	71.8	√		√		√	√	LS	①	9.5	23.7	22.5	25.4	18.9	21
Wu et al., [46]	322	CHN	16.76 ± 0.68	62.4	√				√	√	CSS	②	N/A					20

*Note*. CHN = China, UK = the United Kingdom, CAN = Canada, NZ = New Zealand, KR = South Korea, BE = Belgium, BR = Brazil, PL = Poland, GER = Germany, AUS = Australia, ES = Spain, IRL = Ireland, MX = Mexico; SC = stage of change, PC = process of change, SE = self-efficacy; DB = decisional balance; OV = other variables; PC = precontemplation; *C* = contemplation; *P* = preparation, *A* = action, *M* = maintenance, N/A = not applicable, √ indicates the variable involved in the study; CSS = cross-sectional study, LS = longitudinal study; DA = discriminant analysis, BLRA = dichotomous logistic regression analysis, MRA = multiple regression analysis, HRA = hierarchical regression analysis, CLRA = cross-lagged regression analysis, SEM = structural equation model; ① = forced selection discrete measures, ② = progressive stage measures, ③ = scale continuous measures.

## Data Availability

The data that support the findings of this study are available from the corresponding author upon reasonable request.
